# Ultrasound Evaluation of the Diaphragm in Clinical Anesthesia

**DOI:** 10.1155/2022/2163225

**Published:** 2022-03-03

**Authors:** Yina He, Tiantian Zhao

**Affiliations:** ^1^Department of Anesthesiology, The Second Clinical College of North Sichuan Medical College, Nanchong Central Hospital, Nanchong 637000, Sichuan, China; ^2^Nanchong Central Hospital, The Second Clinical Medical College, North Sichuan Medical College (University), Nanchong 637000, Sichuan, China

## Abstract

When the human body is anesthetized, the human nerve tissue will be greatly affected, which also affects the breathing of the human body. The respiration during anesthesia is a lack of initiative, and the energy efficiency of the diaphragm in the lungs is very important to the safety of anesthesia. In this paper, the application of the ultrasound evaluation of the diaphragm in clinical anesthesia was studied. In this paper, 24 patients who underwent lung examination under medical anesthesia at our hospital were evaluated by the ultrasound vertical mixed echo method. Through patient voluntary selection and consent, 16 patients were examined with B-mode ultrasound and the other 8 patients with M-mode ultrasound to compare the effects of different ultrasounds on diaphragm image quality. In addition, this paper also analyzes the differences between different ultrasounds and the strengths and weaknesses of diaphragmatic ultrasound evaluation in clinical anesthesia. The suggestions of using different ultrasounds in ultrasonic evaluation are given. The study showed that 16 cases of B-mode ultrasound evaluation of the diaphragm obtained ultrasound images which showed a large field of vision, acoustic frequency between 7 and 18 MHz, and thickness difference between 0.35 and 0.52 cm. In 8 patients with the diaphragm evaluated by M-mode ultrasound, the local features of M-mode ultrasound images were clearer than those of B-mode ultrasound images, but the visual field area was smaller, the acoustic frequency was between 10 and 15 MHz, and the thickness difference was between 0.12 and 0.18 cm. Based on the above data, this paper suggests that, in the ultrasonic evaluation of the diaphragm, B-mode ultrasound should be used to check the patients first, and then M-mode ultrasound should be used to check the parts with poor quality so that the accurate diaphragm quality of patients can be obtained in the vast majority of patients.

## 1. Introduction

When anesthetics are applied to the human body, they have a great influence on the nervous tissue of the human body and also affect the breathing of the human body. During anesthesia, the breathing is not smooth. At this time, the energy efficiency of the pulmonary membrane is very important for the safety of people under anesthesia. For example, patients after surgery can be evaluated within 1 hour of mechanical ventilation treatment (60%–70% of the total). Ultrasound evaluation means that it usually needs two to three times of trial failure, which can be successfully evaluated within 7 days after repeated evaluation by clinicians and clinical intervention. Chronic obstructive and restrictive pulmonary disease, heart failure, neuromuscular diseases, and other potential causes often exist in these patients. There is a long time between the complex underlying diseases of patients and the primary diseases leading to acute respiratory failure.

In the study of surgery, BOS thinks that the application of the tubeless technique in the perioperative period of thoracoscopic pulmonary wedge resection is feasible and safe, and it is a less-invasive treatment. However, there is no research on the application of tubeless technology in the treatment of respiratory diseases. This paper fills the gap in this field and provides a reference for further research in the future [1]. Wang et al.'s research showed that the transurethral vaporization of the prostate with the 980 nm/1470 nm dual-wavelength laser under local anesthesia has good efficacy and safety and minimizes the length of hospital stay and hospitalization costs. It is considered that the transurethral vaporization of the prostate with the dual-wavelength laser under local anesthesia can be applied to high-risk patients with BPH [2]. Liu et al. reported that the change of the blood lactate level before and after SBT can be used as a reference index to guide the evaluation time, and the success rate of the evaluation plan based on blood lactate level monitoring is significantly higher [3]. Chen et al.'s study also showed that the blood lactate level is one of the important indicators to evaluate the outcome of patients receiving device ventilation for more than 7 days [4]. Ohsumi et al. proposed that the diaphragm motion parameter, especially diaphragm mobility, is a new widely used evaluation and prediction index, and its prediction effect has been affirmed by some researchers. The blood lactate level is a new indicator that had potential predictive value in recent years [5].

In the study of the diaphragmatic index, Zhang et al. considered that the blood lactate level and diaphragmatic motor function were two relatively independent indexes, and their independent prediction ability did not interfere with each other, and few researchers at home and abroad discussed the predictive value of the combination of the above two indexes in evaluating the outcome [6]. Garutti et al. explored the predictive value of diaphragm motion parameters combined with the blood lactate level before and after SBT in evaluating the outcome in order to find a method that can accurately predict the outcome of patients receiving long-term mechanical ventilation and provide reference for clinical guidance in selecting the evaluation time [7]. Bertani et al. proposed that the use of propofol or inhaled anesthetics during operation did not increase the risk of delirium within 3 days after cardiac surgery. Compared with the propofol group, the incidence of delirium in the inhaled anesthesia group had no significant difference [8]. Watanabe et al. proposed that delirium results are different in different trials due to different evaluation methods and objects. CAM-ICU was used to evaluate delirium. This method is easy to master, and the evaluation time is short. Studies have shown that the sensitivity of this method is 93%, and the specificity is 98% [9]. Qin et al. were induced by intravenous anesthesia. Some studies suggest that propofol is used in combination during anesthesia induction, which has been proved to weaken the potential benefits of inhalation anesthetics and may affect the test results [10]. The time of delirium assessment in the above studies is short, and there are few studies related to delirium mainly due to valve surgery. And there is no use of ultrasound evaluation to detect the pulmonary diaphragm, so the lack of entity detection is not enough to pay attention to the safety of anesthesia.

In this paper, the application of the ultrasound evaluation of the diaphragm in clinical anesthesia was studied. In this paper, 24 cases of patients with pulmonary examination in internal medicine anesthesia in our hospital were evaluated by the ultrasound vertical mixed echo method. In order to compare the effect of different ultrasounds on the image quality of the diaphragm and through the voluntary choice and consent of patients, 16 patients were examined by B-mode ultrasound, and the other 8 patients were examined by M-mode ultrasound. In addition, this paper also analyzes the differences of different ultrasounds and the advantages and disadvantages of the ultrasound evaluation of the diaphragm in clinical anesthesia. The suggestions of using different ultrasounds in ultrasonic evaluation are given.

## 2. Ultrasound Evaluation of the Diaphragm and Sensitivity Factors

### 2.1. Ultrasonic Evaluation Method

When clinicians implement endotracheal intubation, they should think about the timing of patient evaluation at all times. Some guidelines pointed out that when the treatment of patients with primary disease turns, it should be considered to let patients pull out the endotracheal intubation and breathe autonomously [11]. At the same time, some studies have confirmed that nearly half of the ventilation treatment time is used by clinicians to evaluate the timing and implementation process of the evaluation. Removal of endotracheal intubation is not only an important milestone in the process of improving a patient's condition but also poses a considerable risk of complications and failure. Without considering the changes of patients' condition and the pathophysiological changes of evaluation, clinicians rashly decide the time of evaluation and implement the evaluation [12].

In clinical practice, we usually divide the assessment, time required, and difficulty level into simple assessment, ultrasound assessment, and extended assessment. Simple assessment means that patients can complete the assessment of the ventilator and extubation after the first SBT. These kinds of patients usually have no basic lung diseases such as asthma and chronic obstructive pulmonary disease, and their respiratory circulation is relatively stable [13]. Prolonged evaluation refers to the failure of three SBT trials or failure of evaluation after repeated evaluation by clinicians and clinical intervention for more than 7 days after the first SBT [14]. Some patients with prolonged assessment may have dysphagia or respiratory muscle strength problems and other irreversible factors, leading to the need for long-term mechanical ventilation treatment. Screening of evaluation: in some ICUs, senior doctors still make decisions on the evaluation time, but this evaluation method has a high failure rate in all kinds of ICUs. At present, the implementation of daily sedation interruption and SBT trial is encouraged [15].

The application of a rigid bronchoscope in airway diagnosis and treatment has the advantages of simultaneous operation and ventilation, but in terms of the semiclosed state of the whole respiratory circuit and the frequent entry and exit of instruments in the operation process, it cannot effectively avoid the occurrence of air leakage in the circuit [16]. In addition, due to the high responsiveness of the airway itself, the operating space is narrow, and repeated stimulation is easy to cause airway bleeding, edema, spasm, and asphyxia, aggravating the obstruction of ventilation and oxygenation. Therefore, it is very important to find a safe and feasible anesthesia airway management method. In this paper, in order to reduce the occurrence of airway spasm, edema, and other events, both groups were given aminophylline, hormone, and other means as preventive use before operation [17]. During the operation, total intravenous anesthesia was used for induction and maintenance, which effectively avoided the environmental pollution caused by the leakage of inhalation anesthetics. At the same time, Narcotrend continuous EEG monitoring can well guide the maintenance of anesthesia depth and better inhibit the stress reaction caused by the placement of the rigid bronchoscope and the operation process in the airway so that the perioperative hemodynamic indexes of the two groups of patients can be relatively stable as a whole so that the operation can be carried out smoothly without malignant arrhythmia adverse events such as airway spasm, and even surgery termination occurred [18]. Although the heart rate and blood pressure of the two groups fluctuated to a certain extent compared with before operation, the mean arterial pressure was above 65 mmHg, which could better meet the requirements of important tissue and organ perfusion [19]. In addition, it is not difficult to find that the incidence of circulatory instability in the ultrasound evaluation group is obviously higher in a short time. The fluctuation of blood pressure may be related to the changes of intrathoracic pressure and carbon dioxide retention caused by intermittent hand-assisted ventilation. In aeration, there was hypoxemia in the ultrasound evaluation group, and carbon dioxide retention events were significantly higher than those in the S-ultrasound evaluation group. Although intermittent hand control could improve ventilation to some extent, hypercholesterolemia occurred in all patients, and overall pH in the internal environment was not conducive to the management of anesthesia [20]. The reason is that ultrasound evaluation is affected by the Venturi effect and surgical operation. With the increase of injection frequency, the inhaled tidal volume gradually decreases, thus aggravating the obstacle of carbon dioxide discharge. Therefore, it is not suitable for long-term surgical treatment [21]. The S-ultrasound evaluation group was significantly better than the ultrasound evaluation group in maintaining normal oxygenation, without hypoxemia, and internal environment pH and PaCO_2_ were basically maintained at normal levels, so it was more safe and feasible [22]. As a new type of ventilation mode combining normal frequency ventilation with high-frequency ventilation, S-ultrasound evaluation can form a pulse-type inspiratory pressure platform and positive end-expiratory pressure. The pulmonary inspiratory pressure platform produced by normal frequency infusion allows the patient to obtain adequate minute ventilation, improve lung mobilization, promote carbon dioxide release, avoid repeated absorption, and further oxygenate. High-frequency jets can create positive end-expiratory pressure in the lungs. This improves the concentration of alveolar oxygen, helps maintain the mobilization of lung tissue, and promotes oxygen use. In addition, due to the relatively constant airway pressure during the whole ventilation process, the pulmonary vascular resistance is lower, which is more conducive to the improvement of ventilation/blood flow ratio and the prevention of barotrauma [23]. Therefore, it is more recommended for patients with preoperative airway stenosis combined with cardiopulmonary dysfunction; the latter is more conducive to reduce the ventilation dysfunction caused by primary disease. Therefore, as a way of anesthesia management in the perioperative period, through the retrospective analysis of this paper, total intravenous anesthesia is used during the diagnosis and treatment of the rigid trachea, and S-ultrasound evaluation is more conducive to improving the intraoperative oxygenation, maintaining the fluctuation of arterial blood carbon dioxide concentration in the normal range, maintaining the balance of the internal environment, and satisfactorily restraining the injury and stimulation caused by perioperative operation and intubation, while ensuring comfort, it is safe and feasible, which is worthy of clinical recommendation [24].

### 2.2. Ultrasonic Sensitivity Factors and Evaluation Methods

#### 2.2.1. Neurological and Psychological Factors

In the ICU, the environment is quite special, and there are all kinds of noisy machine alarm, rescue voice, day and night, no family accompany, and so on. Patients may be with full of fear, anxiety, and other negative emotions to this environment, which may affect the psychology of patients. A kind of psychoorganic psychological disorder often occurs in critically ill patients, which is called delirium in clinics [25]. The occurrence of delirium increases the risk of prolonged assessment time, as shown in formulas (1)–(3), where *k* is the risk coefficient and *t* is the sexual influence.

(1) $$\begin{array}{c} P\left(b\right)=2n\;\ln\left(\sigma \right)+n\;\ln\left(2\pi \right)+n\left\{\frac{n+\mathrm{tr}\left(S\right)}{n-2-\mathrm{tr}\left(S\right)}\right\}, \end{array}$$

(2) $$\begin{array}{c} S\left(T\right)=K\left(y\left(T-1\right),\ldots ,y\left(t-n\right),u\left(T-d-1\right),\ldots ,u\left(k-d-n\right)\right), \end{array}$$

(3) $$\begin{array}{c} W\left(T\right)=K\left(y\left(T-1\right),u\left(T-d-1\right)\right), \end{array}$$

where *W* is the evaluation function and *D* is the number of iterations. In addition, delirium was associated with respiratory and neurological complications and decreased the success rate of extubation. Relevant scholars want to assist in the evaluation of patients by sunlight exposure. The results show that patients with long sunlight exposure can be more early evaluated.

(4) $$\begin{array}{c} \frac{U}{D}=\sum_{i=1}^{g}\left\{P_{i}|\sum_{j=1}^{k}p_{j}^{\left(i\right)}\right\},\\ U=\left\{\begin{array}{ccc} P_{1}|D,L,f_{2},Q,d,l & P_{2}|f_{1},\mu & P_{3}|N,M,I \end{array}\right\},\\ M=\sum_{S-1}^{U}\sum_{d-1}^{K}f_{s},DV_{s},d. \end{array}$$

However, according to statistics, music therapy has no effect on the evaluation time, but music therapy can improve the heart rate, blood pressure, and coma degree of patients and reduce the dosage of sedative drugs.

#### 2.2.2. Endocrine and Metabolic Factors

There is no relevant evaluation index for this research, but its importance is beyond doubt. We can analyze its impact on assessment (*y*) from two aspects:

(5) $$\begin{array}{c} y_{i}=\beta \left(u_{i},v_{i}\right)+\sum_{j=1}^{p}\beta_{j}\left(u_{i},v_{i}\right)x_{ij}+\varepsilon_{j}\beta_{j},\\ \beta_{j}={\left(X^{T}W_{j}X\right)}^{-1}X^{T}W_{j}Y. \end{array}$$

On the one hand, *W* and *y* are hormone problems. The incidence of hypothyroidism and adrenal insufficiency is low, but it should also be paid attention clinically. On the other hand, in terms of nutrition, the incidence of malnutrition in critically ill patients is very high. The occurrence of malnutrition increased the muscle analysis, resulting in the fatigue of the related respiratory muscles, resulting in the failure of the evaluation.

(6) $$\begin{array}{c} R_{\mathrm{ikjl}}=\left\{\begin{array}{cc} \frac{n}{\Delta_{\mathrm{ikjl}}}\sqrt{\sum_{s=1}^{n}{\left(x_{\mathrm{ik}}\left(\varepsilon \right)-x_{\mathrm{jl}}\left(\varepsilon \right)\right)}^{2}\Delta_{\mathrm{ikjl}}\left(\varepsilon \right)}, & \Delta_{\mathrm{ikjl}}>0,\\ 0, & \Delta_{\mathrm{ikjl}}<0, \end{array}\right.\\ \Delta_{\mathrm{ikjl}}=\sum_{\delta =1}^{n}\Delta_{\mathrm{ikjl}}\left(\varepsilon \right). \end{array}$$

At the same time, the occurrence of malnutrition will cause the decrease of patients' immunity, increase the incidence of hospital pneumonia, and also cause the failure of evaluation.

#### 2.2.3. Iatrogenic Factors

In the whole process of ventilator treatment, clinicians' decision-making is very important. This includes the selection of ventilator parameters and modes in the treatment process, the timing of evaluation, and the interpretation of *N*/*A*, as well as the analysis and treatment of the reasons for the failure of the first evaluation.

(7) $$\begin{array}{c} Q_{\mathrm{ikjl}}\left(\varepsilon \right)=\left\{\begin{array}{cc} 0, & x_{\mathrm{ik}}\left(\varepsilon \right)=\frac{N}{A}\;\mathrm{or}\;x_{\mathrm{jl}}\left(\varepsilon \right)=\frac{N}{A},\\ 1, & x_{\mathrm{ik}}\left(\varepsilon \right)=\frac{N}{A}\;\mathrm{and}\;x_{\mathrm{jl}}\left(\varepsilon \right)=\frac{N}{A}, \end{array}\right.\\ x_{i}=\sum_{j=1}^{n}\omega_{ij}y_{j}-Q_{i}. \end{array}$$

Asynchrony between patients and ventilators is associated with prolonged assessment time and even death. In this paper, rbsi, inferior vena cava variability, and diaphragm displacement were studied from the aspects of evaluation and prediction indexes.

(8) $$\begin{array}{c} \mathrm{AUC}\left(A_{i},A_{j}\right)=\left[\log\left(\frac{\left|x_{A_{i}}-a_{A_{j}}\right|}{Q_{A_{j}}}\right),\;\log\left(\frac{\left|y_{A_{i}}-y_{A_{j}}\right|}{R_{A_{j}}}\right),\;\log\left(\frac{w_{A_{i}}}{R_{A_{j}}}\right),\;\log\left(\frac{h_{A_{i}}}{Q_{A_{j}}}\right)\right]. \end{array}$$

At the same time, this prospective study combined the IVC variability *F* and diaphragm displacement to predict *y*-*j* and compared the IVC variability and diaphragm displacement.

(9) $$\begin{array}{c} y_{i}=f\left(\sum_{j=i}^{k}\omega_{ij}y_{j}-\theta_{i}\right),\;i\neq j. \end{array}$$

Then, combining the two indicators, the prediction accuracy is better than a single indicator, and the application of combined indicators may better guide the evaluation of ventilator ultrasound.

(10) $$\begin{array}{c} H\left(d_{i},w_{j}\right)=H\left(d_{i}\right)H\left(w_{j}|d_{i}\right);P\left(w_{j}|d_{i}\right)=\sum_{k=1}^{K}P\left(w_{j}|z_{k}\right)P\left(z_{k}|d_{i}\right). \end{array}$$

After successful intubation, 15 minutes after one-lung ventilation, the patients were reevaluated according to the oxygenation index, partial pressure of carbon dioxide, mean pulmonary artery pressure, and hemodynamic changes. During the operation, the pulmonary artery was blocked and opened to observe the changes of pulmonary artery pressure and hemodynamics, and the need for ECMO was evaluated.

## 3. Experimental Design

### 3.1. Research Methods

In this paper, the application of the ultrasound evaluation of the diaphragm in clinical anesthesia was studied. In this paper, 24 cases of patients with pulmonary examination in internal medicine anesthesia in our hospital were evaluated by the ultrasound vertical mixed echo method. In order to compare the effect of different ultrasounds on the image quality of the diaphragm and through the voluntary choice and consent of patients, 16 patients were examined by B-mode ultrasound, and the other 8 patients were examined by M-mode ultrasound. In addition, this paper also analyzes the differences of different ultrasounds and the advantages and disadvantages of the ultrasound evaluation of the diaphragm in clinical anesthesia. The suggestions of using different ultrasounds in ultrasonic evaluation are given.

### 3.2. Experimental Content and Detection Design

Extracorporeal membrane oxygenation was performed in 24 patients with respiratory failure, one of which was IPF (preoperative venous arterial placement via the femoral artery and vein). Another patient with covid-19 had advanced pulmonary fibrosis and had intravenous ECMO placed through the femoral and right internal jugular veins. There were 4 patients with mild/moderate tricuspid regurgitation, 1 patient with coronary stenosis, 1 patient with calcified stenosis of the ascending aortic valve, 1 patient with renal insufficiency before operation and received continuous renal replacement therapy regularly, and 1 patient with liver cirrhosis but normal liver function indicated by ultrasound. 18 patients were unable to complete the pulmonary function examination due to various reasons, and 12 out of 13 patients over 50 years old did not undergo coronary CT angiography (CTA) due to emergency operation or illness. The patients with the oxygen bag and nasal catheter were immediately given oxygen with a mask, and the patients with the invasive/noninvasive ventilator were treated with the anesthesia machine to improve hypoxia. Comprehensive monitoring was established, including ECG, invasive blood pressure, oxygen saturation, body temperature, urine volume, end-expiratory carbon dioxide, central venous pressure (CVP), cardiac output (CO), stroke variability, and peripheral vascular resistance. The mean pulmonary artery pressure (mPAP), pulmonary artery systolic pressure (SPAP), and pulmonary capillary wedge pressure (PAWP) were continuously monitored with a floating catheter. Arterial blood gas analysis, coagulation, and platelet function were measured at any time. One patient in the tubeless group had a small amount of pneumothorax after operation, which was considered as the residual gas in the thoracic cavity after operation and then gradually absorbed and disappeared. Therefore, residual gas in the chest cavity should be carefully inhaled at the end of surgery to fully secure lung mobilization and reduce postoperative complications. Compensatory hyperhidrosis is a special complication after thoracoscopic thoracic resection. The mechanism is unclear, and it is mostly considered to be related to the scope of nerve transection. In this study, 3 cases of mild compensatory hyperhidrosis occurred, and the incidence is lower than the previous research level.

The application of the tubeless technology also puts forward higher requirements for the operation team, such as the following: anesthesiologists must be able to change the mode of anesthesia during the operation and solve various emergencies during the operation, such as hypoxemia and hypercapnia. Surgeons must establish accurate evaluation standards and strictly grasp the surgical indications to ensure the safety of patients. Due to the lack of postoperative thoracic drainage, postoperative nursing management is also a great challenge. It is necessary to establish a complete system, such as reasonable selection of surgical patients, perioperative management, formulation of discharge standards, and out-of-hospital follow-up.

## 4. Results and Discussion

### 4.1. Clinical Application of the Ultrasound Evaluation of the Diaphragm

As shown in Figure 1, there is no significant difference in common postoperative complications and compensatory hyperhidrosis between the two groups, but there are still some shortcomings. Most of the patients seeking surgical treatment are moderate and severe patients. Therefore, the number of cases in this study is limited. For patients with obesity, poor lung function, and severe intrathoracic adhesions, the application of this technique is limited, so it is necessary to strictly grasp the surgical indications and contraindications. Respiratory disease is a benign disease. In this paper, some patients with mental and psychological factors were screened out. There may be some bias, so we still need to collect data to carry out large-scale research.

As shown in Figure 2, sufentanil has little effect on heart function, and atracurium cis-benzenesulfonate is Hoffman metabolism, has little effect on the liver and kidney function, and has little histamine release, so it can be safely used in patients with lung transplantation. Dexmedetomidine-combined anesthesia can reduce the inflammatory factors TNF-*α* and IL-6. The serum concentration of 8 can reduce the perioperative inflammatory reaction, oxidative stress, and endoplasmic reticulum stress and reduce the apoptosis of alveolar cells and lung injury. However, propofol can reduce peripheral vascular resistance and myocardial contractility.

As shown in Figure 3, after bronchial anastomosis, the airway was cleaned by suction, and no blood leakage was confirmed by fiberoptic bronchoscopy. The main ventilation mode was pressure control, oxygen concentration was 100%, inspiratory pressure was 18–32 cm, and the summary respiratory rate of anesthesia management in single-center lung transplantation was 12–20 times/min. First, low tidal volume and low airway pressure were used to inflate the transplanted lung slowly and mildly. Then, the volume control mode and appropriate positive end-expiratory pressure were used to gradually adjust. The hypoxic concentration of the new lung should be used as much as possible, which should be lower than 50%.

As shown in Figure 4, it can be seen from Figures 4(a)–4(f) that dexmedetomidine combined with dezocine can provide good sedation and analgesia after lung transplantation, reduce agitation, and contribute to ERAS. In this paper, pure opioid receptor agonists and opioid receptor agonist-antagonists were used for multidisciplinary pain management in order to achieve the goal of individualized analgesia. Postoperative pulmonary infection is still the main cause of early death after lung transplantation. In addition, we found that patients with lung transplantation are older (≥60 years old), have more complications (especially complicated with heart diseases such as coronary artery disease and valve disease), and are in serious condition (patients who need ECMO before operation), and the perioperative mortality is significantly higher, the postoperative mortality is also higher, and the long-term prognosis is poor.

As shown in Figure 5, there were 9 patients with ECMO assistance in this study, of which 2 patients had used ECMO bridging therapy before operation and continued to maintain ECMO assistance during operation. After induction and during one-lung ventilation, 5 patients found that pulmonary artery pressure increased continuously, and circulation was difficult to maintain. Two patients received ECMO after one lung transplantation and found pulmonary arterial pressure increased and hemodynamics changed sharply before the other lung transplantation. The fluid was predominantly colloid as it needed to be as negatively balanced as possible, with the premise of minimizing perfusion.

As shown in Table 1, fluid management follows the principle of injecting fluid in a volume slightly less than the infusion volume while monitoring the cardiac output, peripheral vascular resistance, and stroke fluctuations. The amount of fluid is minimized, and the occurrence of pulmonary edema is reduced. However, these patients have poor tolerance to hypotension. Before induction, they still need to be given 200–300 ml of crystalloid fluid. Intraoperative fluid infusion is mainly colloidal fluid, which should be controlled appropriately before blocking the artery. In order to avoid insufficient volume after opening, ensure effective circulating blood volume, reduce fluid leakage, and reduce the risk of pulmonary edema. It should be noted that when the pulmonary artery is blocked in the second lung transplantation, the incidence of pulmonary edema is increased due to the rapid increase of new lung blood flow. Restrictive infusion and appropriate PEEP can reduce the incidence of pulmonary edema (Table 2).

As shown in Figure 2, in order to avoid insufficient capacity after opening, the colloidal solution should be supplemented appropriately before opening to improve the colloidal osmotic pressure. In patients undergoing double-lung transplantation, limited infusion and appropriate PEEP can reduce pulmonary exudation when the pulmonary artery is blocked in the second lung transplantation. Blood components were supplemented according to intraoperative blood loss, hematocrit, and coagulation indexes.

As shown in Table 3, all patients used esophageal temperature monitoring, temperature-changing blanket, and heater to continuously heat the body surface and the blood transfusion heater to heat the red blood cell components at 38°C. Sevoflurane can reduce the degree of inflammation and oxidation in the lung of patients. It is found that sevoflurane can inhibit TNF-*α* in small airway epithelial cells. Therefore, sevoflurane is an appropriate anesthetic for lung transplantation.

As shown in Figure 6, all patients were managed with multidisciplinary cooperation in perioperative analgesia. Anesthesiologists were equipped with the mechanical analgesia pump. The single patient-controlled analgesia was 0.5 ml/time, and the lock time was 15 min. Intensive care unit (ICU) and thoracic surgeons used corresponding analgesic drugs according to the patient's condition and postoperative pain. The age of all death cases was more than 60 years, including 2 cases with heart valve disease and 1 case with coronary artery stenosis. The mortality of patients over 60 years old was 60% (6/10), and that of patients with heart valve disease or coronary artery disease was 50% (3/6).

As shown in Figure 7, before lung transplantation, patients often suffer from infection, hypoxia, carbon dioxide accumulation, acid-base imbalance, increased pulmonary arterial pressure, and dysfunction of the heart, kidney, liver, and other important organs, and some patients coexist with hypertension and diabetes. It is very important to master the dynamic and up-to-date changes in patient organ function before anesthesia, especially the assessment of cardiopulmonary function related to anesthesia management strategies (including ECMO preparation and selection) and patient prognosis. Etomidate is a better choice for patients with poor cardiopulmonary function.

As shown in Figure 8, the ability of existing drugs to improve pulmonary arterial pressure is limited, so all factors that aggravate pulmonary arterial hypertension should be avoided, and hypotension caused by rapid expansion of blood vessels and myocardial inhibition should be avoided to aggravate pulmonary arterial hypertension. The induction process of all patients in this paper is relatively stable. Once the pulmonary arterial pressure continues to increase and circulation is threatened, ECMO should be used immediately. Any factors that lead to the release of catecholamine may lead to the increase of pulmonary arterial pressure. It is a great challenge for the right and left ventricular function to block and open the pulmonary artery during operation. It is necessary to closely observe the changes of pulmonary artery pressure and right atrial pressure. At present, it is considered that preventive use of ECMO is beneficial. On the contrary, emergency use of ECMO does not improve the prognosis of patients.

As shown in Table 4, the experience of using ECMO is limited, and the timing of using ECMO needs to be further summarized. The expansion of the lung should be slow and mild, the opening of the pulmonary artery should be slow, the oxygen concentration should be as low as possible, in order to maintain the oxygen supply as the premise is to reduce the production of oxygen free radicals, and the oxygen concentration should be less than 50%. Rapid inflation may lead to recruitment pulmonary edema, and it is necessary to prevent hypotension caused by ischemia-reperfusion. Once it occurs, vasoactive drugs should be used to maintain blood pressure and adjust the internal environment to prevent arrhythmia and respiratory and cardiac arrest. Permissive hypercapnia and lung-protective ventilation combined with intraoperative monitoring can improve oxygenation and lung function to the maximum extent.

As shown in Figure 9, one of the 12 patients with double-lung transplantation had poor expansion after opening and increased exudate during the second lung transplantation. Although a series of preventive measures were taken, pulmonary edema could not be avoided. Postoperative pain affects the exercise of respiratory function, suppresses the expectoration of sputum, increases the release of catecholamine, increases the oxygen consumption of the heart and other organs, and increases the risk of cardiovascular and cerebrovascular accidents. Epidural analgesia is beneficial for postoperative respiratory function exercise, but ECMO may help in anticoagulation and increase the risk of epidural hematoma; B-ultrasound-guided thoracic paravertebral nerve block and intercostal nerve block can also be selected as appropriate.

As shown in Figure 10, the ultrasound images obtained from 16 cases of B-mode ultrasound evaluation of the diaphragm showed that the visual field area was large, the acoustic frequency was between 7 and 18 MHz, and the thickness difference was between 0.35 and 0.52 cm. In 8 patients with the diaphragm evaluated by M-mode ultrasound, the local features of M-mode ultrasound images were clearer than those of B-mode ultrasound images, but the visual field area was smaller, the acoustic frequency was between 10 and 15 MHz, and the thickness difference was between 0.12 and 0.18 cm. Based on the above data, this paper suggests that, in the ultrasonic evaluation of the diaphragm, B-mode ultrasound should be used to check the patients first, and then M-mode ultrasound should be used to check the parts with poor quality so that the accurate diaphragm quality of patients can be obtained in the vast majority of patients.

### 4.2. Discussion

Whether oxycodone or morphine is the most commonly used opioid analgesic, in this paper and other large-scale studies, we have observed that the use of oxycodone increased year by year, and the use of morphine decreased year by year (stable), indicating that oxycodone with less adverse reactions, good tolerance, and high safety is expected to become a substitute for morphine. In terms of drug use, the average daily consumption of morphine equivalent in the cancer group was close to that in other studies, while the average daily consumption of morphine equivalent in the noncancer group was lower than that in other studies. In addition, 4.8% of the outpatients who prescribed opioids were noncancer patients, of which 3.3% were noncancer pain patients, which was far lower than other research results. The above results indicate that there are still many obstacles to the use of opioid analgesics in the management of noncancer pain associated with physicians, patients, and families. Doctors' pain and misunderstandings of opioid analgesics lead to inadequate pain management. According to the results of a study, most doctors consider it legal and acceptable to prescribe opioid analgesics for cancer-related pain, but only half of them hold this view for chronic noncancer pain. Many clinicians are reluctant to prescribe opioid analgesics because of the risk of addiction and abuse. In addition, doctors tend to prescribe low-dose opioid analgesics for patients because they are worried about the investigation of opioid analgesics. The drugs are limited to the first or second step analgesics of the three-step analgesic therapy of the World Health Organization. In view of the above problems, pharmacists need to further communicate with doctors to improve their understanding of opioid analgesics, so as to provide adequate pain control for noncancer patients. Secondly, there are obstacles in the use of opioid analgesics such as the fear of adverse drug reactions and addiction and the belief that pain is inevitable and uncontrollable. The adverse reactions of opioid analgesics, such as constipation and nausea, may limit the dosage of opioid analgesics and lead to early withdrawal or insufficient analgesia. 15%–40% of patients receiving opioid analgesics will have nausea and vomiting, and 87% of patients will have constipation. The fear of opioid addiction exists in most patients, their families, and some doctors. In this case, it is necessary to educate the patients and their families about the use of opioids.

## 5. Conclusions

In this paper, 24 cases of patients with pulmonary examination in internal medicine anesthesia in our hospital were evaluated by the ultrasound vertical mixed echo method. The number of samples in this paper is relatively small. In the future, multicenter and large-sample experiments are still needed to prove the predictive value of each index. However, in the data collection stage, whether the measurement of inferior vena cava variability or diaphragm displacement, the measurer must have the qualification of severe ultrasound examination, but there are still subjective factors in the measurement process. In this paper, because the measurement of the left diaphragm displacement is affected by the movement of the heart and lung and the interference of gastrointestinal cavity organs, it is difficult to measure, so the measurement index did not collect the left diaphragm displacement. The limitation of this experiment lies in that there is no dynamic monitoring of multiple time nodes when the measurement time node is SBT 30 min. In the ICU, every clinical intervention and evaluation is the embodiment of clinical experience and wisdom of clinicians. It is expected that there will be better indicators and safer methods to implement the evaluation, so as to benefit patients.

## Figures and Tables

**Figure 1:** Classification of patients interfered by mental and psychological factors.

**Figure 2:** Dexmedetomidine-combined anesthesia can reduce inflammatory factors.

**Figure 3:** Bronchoscopy confirms that there is no bleeding in the anastomosis.

**Figure 4:** Ultrasound evaluation of the diaphragm image (some components in the picture come from the internet and have been authorized by the author).

**Figure 5:** Pulmonary artery pressure found during one-lung ventilation.

**Figure 6:** Disciplinary team of perioperative pain management.

**Figure 7:** Lung transplantation patients often have infections before surgery.

**Figure 8:** Hypotension worsens pulmonary hypertension.

**Figure 9:** Epidural analgesia for postoperative respiratory function.

**Figure 10:** Ultrasound assessment of diaphragm quality results.

**Table 1:** Odds of pulmonary edema.

Item	Oxygen partial pressure	Partial pressure of carbon dioxide	Mean arterial pressure	Diaphragm mobility
Sepsis	2.7	2.81	3.94	3.97
Merge	5.03	2.63	2.04	2.95
Basis	2.73	4.08	2.05	2.76
Disease	4.73	4.04	3.49	4.73
Heart failure	2.06	1.54	2.61	2.12

**Table 2:** Transplant to block the pulmonary artery.

Item	Success	Failure	Primary disease	Respiratory failure	Heart failure
Merge	2.54	2.08	2.23	2.92	3.85
Basis	5.85	4.95	5.77	3.19	4.54
Disease	3.31	1.43	5.96	1.69	5.57
Hypertension	3.13	2.63	1.16	2.96	4.01
Diabetes	2.48	1.49	6.03	6.82	5.84

**Table 3:** The degree of inflammation and oxidation in the patient lungs.

Item	Wall thickness	Groove	Beam angle	Depth of the incident	Data collection
Basis	2.7	2.81	3.94	3.97	2.88
Disease	5.03	2.63	2.04	2.95	2
Hypertension	2.73	4.08	2.05	2.76	3.64
Diabetes	4.73	4.04	3.49	4.73	2.63
Coronary heart	2.06	1.54	2.61	2.12	3.99
COPD	1.65	1.3	4.46	1.52	3.24

**Table 4:** Production of oxygen free radicals.

Item	Value of heart rate (beats/min)	Respiration rate (times/min)	Oxygen partial pressure	Partial pressure of carbon dioxide
TCG	0.99	0.52	0.21	1.33
Failure	5.85	4.95	5.77	3.19
Primary disease	3.31	1.43	5.96	1.69
Respirator	3.13	2.63	1.16	2.96

## Data Availability

We do not have permission to share the data from the data provider.

## References

[1] Bos S., Vos R., van Raemdonck D. E., Verleden G. M. (2020). Survival in adult lung transplantation: where are we in 2020?. *Current Opinion in Organ Transplantation*.

[2] Wang Q., Jiang X. L., Qin G. W., Wang X., Wang Z. (2017). Effect of anesthetic factors on perioperative inflammatory responses in bilateral lung transplantation: advantages of dexmete-tomidine-based anesthesia. *Chinese Journal of Anesthesiology*.

[3] Liu Z., Meng Y., Miao Y., Yu L., Yu Q. (2020). Propofol reduces renal ischemia/reperfusion-induced acute lung injury by stimulating sirtuin 1 and inhibiting pyroptosis. *Aging*.

[4] Chen C.-Y., Tsai Y.-F., Huang W.-J., Chang S.-H., Hwang T.-L. (2018). Propofol inhibits endogenous formyl peptide-induced neutrophil activation and alleviates lung injury. *Free Radical Biology and Medicine*.

[5] Ohsumi A., Marseu K., Slinger P. (2017). Sevoflurane attenuates ischemia-reperfusion injury in a Rat Lung Transplantation model. *The Annals of Thoracic Surgery*.

[6] Zhang L., Li D. H., Guo X. B. (2020). Research progress of drugs that attenuate oxidative stress in lung ischemia reperfusion injury. *Medical Journal of Wuhan University*.

[7] Garutti I., Gonzalez-Moraga F., Sanchez-Pedrosa G. (2019). The effect of anesthetic preconditioning with sevoflurane on intracellular signal-transduction pathways and apoptosis, in a lung autotransplant experimental model. *Brazilian Journal of Anesthesiology (English Edition)*.

[8] Bertani A., Miceli V., De Monte L. (2021). Donor preconditioning with inhaled sevoflurane mitigates the effects of ischemia-reperfusion injury in a swine model of lung transplantation. *BioMed Research International*.

[9] Watanabe K., Iwahara C., Nakayama H. (2019). Sevoflurane suppresses tumour necrosis factor-*α*-induced inflammatory responses in small airway epithelial cells afteranoxia/reoxygenation. *British Journal of Anaesthesia*.

[10] Qin Z., Yang Y. G., Wang Z. P. (2019). Anesthetic management of 80 cases of bilateral sequential lung transplantation. *Journal of Clinical Pulmonary Medicine*.

[11] Hu C. X., Wang Z. P., Xu B. (2019). Perioperative management of lung transplantation. *Chinese Journal of Anesthesiology*.

[12] Hu C. X., Xu B., Wang Z. P., Yang Z. P., Wu J., Chen J. (2017). Perioperative anaesthetic management of bilateral lung transplantation for idiopathic pulmonary arterial hypertension. *The Journal of Clinical Anesthesiology*.

[13] Tang F. D., Li M. X. (2012). Anesthetic management for lung transplantation. *Hainan Medical Journal*.

[14] Hu C. X., Wang Z. P., Xu B. (2019). Anesthetic management of pulmonary arterial hypertension for lung transplantation. *Chinese Journal of Organ Transplantation*.

[15] Li X. S., Chen J. Y., Yu H. Z. (2020). Preliminary efficacy comparison of lung transplantation between VA and VV bypass types of extracorporeal membrane oxygenation. *Chinese Journal of Organ Transplantation*.

[16] Wang Q., Jiang X. L., Qin G. W., Wang X., Wang Z. (2018). Efficacy of dexmedetomidine mixed with sufentanil for patient-controlled intravenous analgesia after double lung transplantation. *Chinese Journal of Anesthesiology*.

[17] Jiang S. Y., Xu H. Y., Wang D. P. (2018). Analgesic and sedative efficacy of decozine combined with dexmedetomidine in patients after lung transplantation. *Guang-dong Medicine*.

[18] Cui F., Liu J., Li S. (2016). Tubeless video-assisted thoracoscopic surgery (VATS) under non-intubated, intravenous anesthesia with spontaneous ventilation and no placement of chest tube postoperatively. *Journal of Thoracic Disease*.

[19] He J., Liu J., Zhu C. (2019). Expert consensus on tubeless video-assisted thoracoscopic surgery (Guangzhou). *Journal of Thoracic Disease*.

[20] Hornberger J., Grimes K., Naumann M. (2019). Recognition, diagnosis, and treatment of primary focal hyperhidrosis. *Joint American Academy of Dermatology*.

[21] Nawrocki S., Cha J. (2019). The etiology, diagnosis, and management of hyperhidrosis: a comprehensive review. *Journal of the American Academy of Dermatology*.

[22] Chen J., Liu Y., Yang J. (2019). Endoscopic thoracic sympathicotomy for primary palmar hyperhidrosis: a retrospective multicenter study in China. *Surgery*.

[23] Lai F. C., Tu Y. R., Li Y. P. (2019). Nation wide epidemiological survey of primary palmar hyperhidrosis in the people’s Republic of China. *Clinical Autonomic Research*.

[24] Kamberov Y. G., Wang S., Tan J. (2019). Modeling recent human evolution in mice by expression of a selected EDAR variant. *Cell*.

[25] Liu C. Y., Hsu P. K., Leong K. I., Ting C., Tsou M. (2020). Is tubeless uniportal video-assisted thoracic surgery for pulmonary wedge resection a safe procedure?. *European Journal of Cardio-Thoracic Surgery*.

